The article "{μ-6,6′-Dimeth­oxy-2,2′-[ethane-1,2-diylbis(nitrilo­methyl­idyne)]diphenolato}-μ-nitrato-dinitratoholmium(III)zinc(II)" was retracted in 2010. Reasons: fabricated or falsified data; errors in the data.

# {μ-6,6′-Dimeth­oxy-2,2′-[ethane-1,2-diylbis(nitrilo­methyl­idyne)]diphenolato}-μ-nitrato-dinitratoholmium(III)zinc(II)

**DOI:** 10.1107/S1600536808013743

**Published:** 2008-05-14

**Authors:** Yi-An Xiao, Yan Sui, Xiu-Guang Yi, Jian-Hong Wu, Li-Ping Zhang

**Affiliations:** a College of Life Science, JingGangShan University, 343009 Ji’an, JiangXi, People’s Republic of China; b JiangXi Province Key Laboratory of Coordination Chemistry, College of Chemistry & Chemical Engineering, JingGangShan University, 343009 Ji’an, JiangXi, People’s Republic of China

## Abstract

In the title heteronuclear Zn^II^–Ho^III^ complex (systematic name: {μ-6,6′-dimeth­oxy-2,2′-[ethane-1,2-diylbis(nitrilo­methyl­idyne)]diphenolato-1κ^4^ *O* ^1^,*O* ^1′^,*O* ^6^,*O* ^6′^:2κ^4^ *O* ^1^,*N*,*N*′,*O* ^1′^)-μ-nitrato-1:2κ^2^ *O*:*O*′-dinitrato-1κ^4^ *O*,*O*′-holmium(III)zinc(II)), [HoZn(C_18_H_18_N_2_O_4_)(NO_3_)_3_], with the hexa­dentate Schiff base compartmental ligand *N*,*N*′-bis­(3-methoxy­salicyl­idene)ethyl­enediamine (H_2_ *L*), the Ho and Zn atoms are triply bridged by two phenolate O atoms of the Schiff base ligand and one nitrate ion. The five-coordinate Zn atom is in a square-pyramidal geometry with the donor centers of two imine N atoms, two phenolate O atoms and one of the bridging nitrate O atoms. The Ho^III^ center has a ninefold coordination environment of O atoms, involving the phenolate O atoms, two meth­oxy O atoms, two O atoms from two nitrate ions and one from the bridging nitrate ion. Weak inter­molecular C—H⋯O inter­actions generate a two-dimensional double-layer structure.

## Related literature

For related literature, see: Baggio *et al.* (2000 ▶); Caravan *et al.* (1999 ▶); Edder *et al.* (2000 ▶); Knoer *et al.* (2005 ▶); Sui *et al.* (2006 ▶, 2007 ▶).

## Experimental

### 

#### Crystal data

[HoZn(C_18_H_18_N_2_O_4_)(NO_3_)_3_]
*M* *_r_* = 742.67
Monoclinic,
*a* = 10.694 (4) Å
*b* = 16.481 (7) Å
*c* = 14.921 (6) Å
β = 99.667 (6)°
*V* = 2592.4 (18) Å^3^
*Z* = 4
Mo *K*α radiation
μ = 4.03 mm^−1^
*T* = 293 (2) K
0.16 × 0.16 × 0.10 mm

#### Data collection

Bruker APEXII area-detector diffractometer
Absorption correction: multi-scan (*SADABS*; Bruker, 2004 ▶) *T*_min_ = 0.565, *T*_max_ = 0.689
15217 measured reflections
4499 independent reflections
3377 reflections with *I* > 2σ(*I*)
*R*_int_ = 0.037

#### Refinement

*R*[*F* ^2^ > 2σ(*F* ^2^)] = 0.034
*wR*(*F* ^2^) = 0.093
*S* = 1.02
4499 reflections
345 parameters
2 restraints
H-atom parameters constrained
Δρ_max_ = 0.60 e Å^−3^
Δρ_min_ = −1.18 e Å^−3^

### 

Data collection: *APEX2* (Bruker, 2004 ▶); cell refinement: *APEX2*; data reduction: *APEX2*; program(s) used to solve structure: *SHELXS97* (Sheldrick, 2008 ▶); program(s) used to refine structure: *SHELXL97* (Sheldrick, 2008 ▶); molecular graphics: *APEX2*; software used to prepare material for publication: *APEX2* and *publCIF* (Westrip, 2008 ▶).

## Supplementary Material

Crystal structure: contains datablocks I, global. DOI: 10.1107/S1600536808013743/at2567sup1.cif

Structure factors: contains datablocks I. DOI: 10.1107/S1600536808013743/at2567Isup2.hkl

Additional supplementary materials:  crystallographic information; 3D view; checkCIF report

## Figures and Tables

**Table 1:** Selected bond lengths (Å)

Ho1—O1	2.293 (3)
Ho1—O2	2.298 (3)
Ho1—O3	2.604 (4)
Ho1—O4	2.604 (4)
Ho1—O6	2.323 (4)
Ho1—O8	2.448 (4)
Ho1—O9	2.481 (4)
Ho1—O11	2.430 (4)
Ho1—O12	2.468 (4)
Zn1—O1	2.005 (4)
Zn1—O2	2.022 (3)
Zn1—O5	1.979 (4)
Zn1—N1	2.047 (4)
Zn1—N2	2.021 (5)

**Table 2:** Hydrogen-bond geometry (Å, °)

*D*—H⋯*A*	*D*—H	H⋯*A*	*D*⋯*A*	*D*—H⋯*A*
C5—H5⋯O11^i^	0.93	2.45	3.377 (7)	174
C10—H10*A*⋯O13^ii^	0.97	2.54	3.483 (8)	165

Symmetry codes: (i) ; (ii) .

## supplementary crystallographic information

### Comment

The potential applications of trivalent lanthanide complexes as contrast agent for magnetic resonance imaging and stains for fluorescence imaging have prompted considerable interest in the preparation, magnetic and optical properties of 3d-4f hetorometallic dinuclear complexes (Baggio *et al.*, 2000; Caravan *et al.*, 1999; Edder *et al.*, 2000; Knoer *et al.*, 2005). As part of our investigations into the structure and applications of 3d-4f hetorometallic Schiff base complexes (Sui *et al.* 2006; Sui *et al.* 2007), we report here the synthesis and X-ray crystal structure analysis of the title complex, (I), a new Zn^II^—Ho^III^ complex with salen-type Schiff base *N*,*N*'-bis(3-methoxysalicylidene) ethylenediamine (H_2_L).

Complex (I) crystallizes in the space group *P*2_1_/*n*, with zinc and holmium triply bridged by two phenolate O atoms provided by the Schiff base ligand and one nitrate ion. The inner salen-type cavity is occupied by zinc(II), while holmium(III) is present in the open and larger portion of the dinucleating compartmental Schiff base ligand.

The Ho^III^ center has a ninefold coordination environment of O atoms, involving the phenolate O atoms, two methoxy O atoms, two O atoms from two nitrate ions and one from the bridging nitrate ion. The four kinds of Ho—O bond distances are significantly different, the longest being the Ho—*O *(methoxy) separations and the shortest being the Ho—O (phenolate).

The Zn^II^ is in a square-pyramidal geometry and is five-coordinated by two imine N atoms, two phenolate O atoms and one of the bridging nitrate O atoms. The Zn atom is 0.6067 (4) Å below the mean N_2_O_2_ plane with an average deviation from the plane of 0.0380 (3) Å, which construct the bottom of square-pyramid. The Zn—O5 (bridging nitrate) separation is 1.979 (4) Å and the angles of this Zn—O vector with the Zn—N or Zn—O bonds lie between 102.5 (4)° and 112.6 (4)°, which suggesting that the Zn^II^ is in a slightly distorted square-pyramidal conformation.

Adjacent molecules are held together by weak interactions [C5(H5)···O11^i ^= 3.377 (7) Å and C10(H10A)···O13^ii ^= 3.483 (8) Å; symmetry codes: (i) -1/2 + *x*, 1/2 - *y*, 1/2 + *z*; (ii) 1 - *x*, -*y*, 2 - *z*]. These link the molecules into a two-dimensional double layer structure (Fig 2).

### Experimental

H_2_L was prepared by the 2:1 condensation of 3-methoxysalicylaldehyde and ethylenediamine in methanol. Complex (I) was obtained by the treatment of zinc(II) acetate dihydrate (0.188 g, 1 mmol) with H_2_L (0.328 g, 1 mmol) in methanol solution (80 ml) under reflux for 3 h and then for another 3 h after the addition of holmium(III) nitrate hexahydrate (0.459 g, 1 mmol). The reaction mixture was cooled and the resulting precipitate was filtered off, washed with diethyl ether and dried *in vacuo*. Single crystals of (I) suitable for X-ray analysis were obtained by slow evaporation at room temperature of a methanol solution. Analysis calculated for C_18_H_18_HoN_5_O_13_Zn: C 29.11 H 2.44, Ho 22.21, N 9.43, Zn 8.80%; found: C 29.20, H 2.45, Ho 22.30, N 9.50, Zn 8.90%. IR (KBr, cm^-1^): 1640 (C=N), 1386,1490 (nitrate).

### Refinement

The H atoms were positioned geometrically and treated as riding on their parent atoms, with C—H distances of 0.93 (aromatic), 0.97 (methylene) and 0.96 Å (methyl), and with *U*_iso_(H) = 1.5*U*_eq_(C) for methyl H atoms and 1.2*U*_eq_(C) for other H atoms. The main directions of movement of covalently bonded atoms N3, O5 and O6 are enforced to be the same.

### Crystal data

**Table:**

[HoZn(C_18_H_18_N_2_O_4_)(NO_3_)_3_]	*F*_000_ = 1448
*M**_r_* = 742.67	*D*_x_ = 1.903 Mg m^−^^3^
Monoclinic, *P*2_1_/*n*	Mo *K*α radiation λ = 0.71073 Å
Hall symbol: -P 2yn	Cell parameters from 5632 reflections
*a* = 10.694 (4) Å	θ = 2.2–25.3º
*b* = 16.481 (7) Å	µ = 4.03 mm^−^^1^
*c* = 14.921 (6) Å	*T* = 293 (2) K
β = 99.667 (6)º	Block, yellow
*V* = 2592.4 (18) Å^3^	0.16 × 0.16 × 0.10 mm
*Z* = 4	

### Data collection

**Table:**

Bruker APEXII area-detector diffractometer	4499 independent reflections
Radiation source: fine-focus sealed tube	3377 reflections with *I* > 2σ(*I*)
Monochromator: graphite	*R*_int_ = 0.037
*T* = 293(2) K	θ_max_ = 25.0º
φ and ω scans	θ_min_ = 2.2º
Absorption correction: multi-scan(SADABS; Bruker, 2004)	*h* = −12→12
*T*_min_ = 0.565, *T*_max_ = 0.689	*k* = −19→19
15217 measured reflections	*l* = −17→17

### Refinement

**Table:**

Refinement on *F*^2^	Secondary atom site location: difference Fourier map
Least-squares matrix: full	Hydrogen site location: inferred from neighbouring sites
*R*[*F*^2^ > 2σ(*F*^2^)] = 0.034	H-atom parameters constrained
*wR*(*F*^2^) = 0.093	*w* = 1/[σ^2^(*F*_o_^2^) + (0.0558*P*)^2^ + 0.1192*P*] where *P* = (*F*_o_^2^ + 2*F*_c_^2^)/3
*S* = 1.02	(Δ/σ)_max_ < 0.001
4499 reflections	Δρ_max_ = 0.61 e Å^−^^3^
345 parameters	Δρ_min_ = −1.18 e Å^−^^3^
2 restraints	Extinction correction: none
Primary atom site location: structure-invariant direct methods	

### Special details

**Table:**

Geometry. All e.s.d.'s (except the e.s.d. in the dihedral angle between two l.s. planes) are estimated using the full covariance matrix. The cell e.s.d.'s are taken into account individually in the estimation of e.s.d.'s in distances, angles and torsion angles; correlations between e.s.d.'s in cell parameters are only used when they are defined by crystal symmetry. An approximate (isotropic) treatment of cell e.s.d.'s is used for estimating e.s.d.'s involving l.s. planes.
Refinement. Refinement of *F*^2^ against ALL reflections. The weighted *R*-factor *wR* and goodness of fit *S* are based on *F*^2^, conventional *R*-factors *R* are based on *F*, with *F* set to zero for negative *F*^2^. The threshold expression of *F*^2^ > σ(*F*^2^) is used only for calculating *R*-factors(gt) *etc*. and is not relevant to the choice of reflections for refinement. *R*-factors based on *F*^2^ are statistically about twice as large as those based on *F*, and *R*- factors based on ALL data will be even larger.

### Fractional atomic coordinates and isotropic or equivalent isotropic displacement parameters (Å^2^)

**Table:**

	*x*	*y*	*z*	*U*_iso_*/*U*_eq_	
Ho1	0.36187 (2)	0.109293 (15)	0.723858 (16)	0.04439 (11)	
Zn1	0.21999 (6)	0.03550 (4)	0.88927 (4)	0.04303 (17)	
O1	0.2906 (4)	0.1419 (2)	0.8559 (2)	0.0493 (9)	
O12	0.5712 (4)	0.1290 (3)	0.8198 (3)	0.0640 (12)	
O2	0.3521 (4)	−0.0016 (2)	0.8158 (2)	0.0497 (9)	
O4	0.4894 (3)	−0.0201 (2)	0.6956 (2)	0.0495 (9)	
C17	0.4119 (5)	−0.0722 (3)	0.8204 (3)	0.0413 (12)	
O8	0.2843 (4)	0.1975 (2)	0.5945 (2)	0.0582 (10)	
N4	0.2806 (5)	0.1437 (3)	0.5329 (4)	0.0624 (14)	
O6	0.1491 (4)	0.0740 (3)	0.6881 (3)	0.0613 (11)	
C3	0.2935 (6)	0.3590 (4)	0.8767 (4)	0.0567 (15)	
H3	0.3175	0.4036	0.8452	0.068*	
N5	0.6224 (5)	0.1590 (4)	0.7564 (4)	0.0659 (15)	
O5	0.0581 (3)	0.0283 (2)	0.8031 (3)	0.0543 (10)	
C16	0.4896 (5)	−0.0846 (3)	0.7542 (4)	0.0460 (13)	
O9	0.3274 (4)	0.0751 (3)	0.5596 (3)	0.0624 (11)	
C2	0.3092 (5)	0.2813 (3)	0.8465 (3)	0.0448 (13)	
C12	0.4039 (5)	−0.1325 (3)	0.8854 (4)	0.0457 (13)	
N3	0.0556 (5)	0.0490 (3)	0.7206 (4)	0.0695 (14)	
O11	0.5537 (4)	0.1634 (3)	0.6792 (3)	0.0612 (11)	
O10	0.2350 (6)	0.1567 (3)	0.4552 (3)	0.107 (2)	
N1	0.1978 (4)	0.0839 (3)	1.0120 (3)	0.0506 (12)	
N2	0.2494 (4)	−0.0675 (3)	0.9634 (3)	0.0488 (11)	
C11	0.3278 (5)	−0.1246 (4)	0.9578 (4)	0.0513 (15)	
H11	0.3374	−0.1641	1.0030	0.062*	
C7	0.2716 (5)	0.2135 (3)	0.8916 (3)	0.0428 (12)	
C8	0.1985 (5)	0.1588 (4)	1.0310 (4)	0.0573 (16)	
H8	0.1823	0.1728	1.0884	0.069*	
C10	0.1754 (6)	−0.0615 (4)	1.0385 (4)	0.0590 (16)	
H10A	0.2017	−0.1037	1.0830	0.071*	
H10B	0.0859	−0.0688	1.0151	0.071*	
C6	0.2222 (5)	0.2248 (3)	0.9720 (4)	0.0500 (14)	
C18	0.5665 (6)	−0.0292 (4)	0.6251 (4)	0.0638 (17)	
H18A	0.6543	−0.0328	0.6524	0.096*	
H18B	0.5544	0.0168	0.5852	0.096*	
H18C	0.5421	−0.0777	0.5910	0.096*	
C5	0.2056 (6)	0.3045 (4)	1.0014 (4)	0.0631 (17)	
H5	0.1699	0.3130	1.0533	0.076*	
O13	0.7311 (5)	0.1830 (4)	0.7710 (4)	0.112 (2)	
C4	0.2412 (7)	0.3697 (4)	0.9550 (4)	0.0643 (18)	
H4	0.2302	0.4219	0.9762	0.077*	
C15	0.5530 (6)	−0.1572 (4)	0.7500 (4)	0.0569 (15)	
H15	0.6023	−0.1659	0.7052	0.068*	
C9	0.1972 (6)	0.0203 (4)	1.0823 (4)	0.0612 (17)	
H9A	0.1307	0.0317	1.1174	0.073*	
H9B	0.2777	0.0205	1.1234	0.073*	
C14	0.5419 (6)	−0.2169 (4)	0.8140 (5)	0.0701 (19)	
H14	0.5833	−0.2662	0.8113	0.084*	
C13	0.4716 (6)	−0.2043 (4)	0.8802 (4)	0.0623 (17)	
H13	0.4683	−0.2446	0.9235	0.075*	
O7	−0.0708 (6)	0.0407 (5)	0.6557 (5)	0.142 (3)	
O3	0.3629 (4)	0.2616 (2)	0.7706 (2)	0.0502 (9)	
C1	0.4246 (7)	0.3260 (4)	0.7307 (4)	0.0661 (17)	
H1A	0.3638	0.3673	0.7090	0.099*	
H1B	0.4611	0.3051	0.6808	0.099*	
H1C	0.4903	0.3486	0.7755	0.099*	

### Atomic displacement parameters (Å^2^)

**Table:**

	*U*^11^	*U*^22^	*U*^33^	*U*^12^	*U*^13^	*U*^23^
Ho1	0.05102 (19)	0.04515 (17)	0.04112 (16)	0.00162 (12)	0.01960 (11)	0.00255 (11)
Zn1	0.0470 (4)	0.0447 (4)	0.0411 (3)	−0.0003 (3)	0.0182 (3)	0.0028 (3)
O1	0.067 (3)	0.036 (2)	0.052 (2)	−0.0004 (19)	0.034 (2)	−0.0054 (18)
O12	0.050 (2)	0.091 (3)	0.053 (2)	−0.010 (2)	0.0144 (19)	0.013 (2)
O2	0.064 (3)	0.042 (2)	0.051 (2)	0.0077 (19)	0.0327 (19)	0.0102 (17)
O4	0.060 (2)	0.048 (2)	0.047 (2)	0.0107 (19)	0.0264 (18)	0.0023 (18)
C17	0.035 (3)	0.037 (3)	0.051 (3)	0.003 (2)	0.006 (2)	0.000 (3)
O8	0.081 (3)	0.049 (2)	0.045 (2)	0.013 (2)	0.014 (2)	0.0020 (19)
N4	0.076 (4)	0.063 (3)	0.053 (3)	0.018 (3)	0.024 (3)	0.004 (3)
O6	0.058 (3)	0.074 (3)	0.052 (2)	−0.010 (2)	0.0101 (18)	0.007 (2)
C3	0.068 (4)	0.039 (3)	0.060 (4)	0.001 (3)	0.003 (3)	0.001 (3)
N5	0.056 (4)	0.079 (4)	0.068 (4)	−0.008 (3)	0.024 (3)	0.003 (3)
O5	0.047 (2)	0.055 (2)	0.064 (2)	−0.0028 (19)	0.0182 (19)	0.0082 (19)
C16	0.044 (3)	0.047 (3)	0.048 (3)	0.004 (3)	0.010 (2)	−0.002 (3)
O9	0.088 (3)	0.055 (3)	0.047 (2)	0.015 (2)	0.021 (2)	0.000 (2)
C2	0.053 (3)	0.035 (3)	0.045 (3)	0.003 (3)	0.004 (2)	−0.001 (2)
C12	0.041 (3)	0.044 (3)	0.053 (3)	−0.002 (3)	0.009 (3)	0.002 (3)
N3	0.065 (3)	0.072 (4)	0.072 (3)	−0.007 (3)	0.015 (3)	0.010 (3)
O11	0.060 (3)	0.079 (3)	0.048 (2)	−0.007 (2)	0.021 (2)	0.014 (2)
O10	0.154 (5)	0.118 (5)	0.043 (3)	0.058 (4)	0.003 (3)	0.004 (3)
N1	0.052 (3)	0.062 (3)	0.044 (3)	−0.005 (2)	0.024 (2)	−0.001 (2)
N2	0.047 (3)	0.052 (3)	0.049 (3)	0.001 (2)	0.015 (2)	0.010 (2)
C11	0.049 (4)	0.053 (4)	0.050 (3)	−0.007 (3)	0.003 (3)	0.011 (3)
C7	0.043 (3)	0.049 (3)	0.037 (3)	−0.001 (3)	0.008 (2)	−0.012 (3)
C8	0.055 (4)	0.078 (5)	0.044 (3)	0.000 (3)	0.025 (3)	−0.013 (3)
C10	0.056 (4)	0.070 (4)	0.055 (3)	−0.006 (3)	0.021 (3)	0.024 (3)
C6	0.058 (4)	0.048 (3)	0.045 (3)	0.001 (3)	0.012 (3)	−0.013 (3)
C18	0.071 (4)	0.068 (4)	0.063 (4)	0.011 (3)	0.040 (3)	0.003 (3)
C5	0.069 (4)	0.072 (5)	0.051 (3)	0.010 (4)	0.016 (3)	−0.022 (3)
O13	0.064 (3)	0.173 (6)	0.100 (4)	−0.036 (4)	0.021 (3)	0.026 (4)
C4	0.085 (5)	0.051 (4)	0.056 (4)	0.013 (4)	0.009 (3)	−0.016 (3)
C15	0.053 (4)	0.055 (4)	0.065 (4)	0.014 (3)	0.018 (3)	−0.007 (3)
C9	0.065 (4)	0.077 (5)	0.046 (3)	0.000 (3)	0.023 (3)	0.007 (3)
C14	0.067 (4)	0.046 (4)	0.102 (5)	0.021 (3)	0.025 (4)	0.006 (4)
C13	0.062 (4)	0.045 (4)	0.080 (4)	0.009 (3)	0.013 (3)	0.020 (3)
O7	0.099 (5)	0.175 (7)	0.138 (6)	−0.011 (5)	−0.026 (4)	−0.001 (5)
O3	0.067 (3)	0.038 (2)	0.049 (2)	−0.0051 (19)	0.0216 (18)	0.0003 (18)
C1	0.092 (5)	0.048 (4)	0.063 (4)	−0.013 (4)	0.026 (3)	0.005 (3)

### Geometric parameters (Å, °)

**Table:**

Ho1—O1	2.293 (3)	C2—C7	1.398 (7)
Ho1—O2	2.298 (3)	C12—C13	1.396 (8)
Ho1—O3	2.604 (4)	C12—C11	1.463 (8)
Ho1—O4	2.604 (4)	N3—O7	1.531 (8)
Ho1—O6	2.323 (4)	N1—C8	1.267 (8)
Ho1—O8	2.448 (4)	N1—C9	1.484 (7)
Ho1—O9	2.481 (4)	N2—C11	1.273 (7)
Ho1—O11	2.430 (4)	N2—C10	1.480 (6)
Ho1—O12	2.468 (4)	C11—H11	0.9300
Zn1—O1	2.005 (4)	C7—C6	1.401 (7)
Zn1—O2	2.022 (3)	C8—C6	1.449 (8)
Zn1—O5	1.979 (4)	C8—H8	0.9300
Zn1—N1	2.047 (4)	C10—C9	1.498 (9)
Zn1—N2	2.021 (5)	C10—H10A	0.9700
O1—C7	1.324 (6)	C10—H10B	0.9700
O12—N5	1.269 (6)	C6—C5	1.406 (8)
O2—C17	1.325 (6)	C18—H18A	0.9600
O4—C16	1.376 (6)	C18—H18B	0.9600
O4—C18	1.449 (6)	C18—H18C	0.9600
C17—C12	1.402 (7)	C5—C4	1.367 (9)
C17—C16	1.408 (7)	C5—H5	0.9300
O8—N4	1.273 (6)	C4—H4	0.9300
N4—O10	1.199 (6)	C15—C14	1.390 (9)
N4—O9	1.272 (6)	C15—H15	0.9300
O6—N3	1.251 (6)	C9—H9A	0.9700
C3—C2	1.379 (8)	C9—H9B	0.9700
C3—C4	1.389 (9)	C14—C13	1.355 (9)
C3—H3	0.9300	C14—H14	0.9300
N5—O13	1.213 (7)	C13—H13	0.9300
N5—O11	1.260 (6)	O3—C1	1.431 (6)
O5—N3	1.274 (6)	C1—H1A	0.9600
C16—C15	1.382 (8)	C1—H1B	0.9600
C2—O3	1.390 (6)	C1—H1C	0.9600
			
O1—Ho1—O2	67.54 (12)	C15—C16—C17	120.6 (5)
O1—Ho1—O6	78.56 (14)	N4—O9—Ho1	95.4 (3)
O2—Ho1—O6	78.26 (14)	C3—C2—O3	124.9 (5)
O1—Ho1—O11	124.55 (14)	C3—C2—C7	121.6 (5)
O2—Ho1—O11	125.51 (14)	O3—C2—C7	113.4 (4)
O6—Ho1—O11	150.31 (13)	C13—C12—C17	118.0 (5)
O1—Ho1—O8	114.92 (13)	C13—C12—C11	118.3 (5)
O2—Ho1—O8	154.15 (14)	C17—C12—C11	123.7 (5)
O6—Ho1—O8	77.22 (14)	O6—N3—O5	125.0 (5)
O11—Ho1—O8	75.84 (14)	O6—N3—O7	117.5 (5)
O1—Ho1—O12	82.58 (14)	O5—N3—O7	117.4 (5)
O2—Ho1—O12	83.46 (14)	N5—O11—Ho1	96.7 (3)
O6—Ho1—O12	157.61 (13)	C8—N1—C9	122.1 (5)
O11—Ho1—O12	52.07 (13)	C8—N1—Zn1	125.6 (4)
O8—Ho1—O12	122.24 (14)	C9—N1—Zn1	111.8 (4)
O1—Ho1—O9	152.44 (15)	C11—N2—C10	122.7 (5)
O2—Ho1—O9	113.29 (14)	C11—N2—Zn1	129.0 (4)
O6—Ho1—O9	74.88 (14)	C10—N2—Zn1	107.7 (4)
O11—Ho1—O9	78.74 (14)	N2—C11—C12	124.6 (5)
O8—Ho1—O9	51.77 (13)	N2—C11—H11	117.7
O12—Ho1—O9	124.92 (14)	C12—C11—H11	117.7
O1—Ho1—O4	126.16 (12)	O1—C7—C2	116.2 (4)
O2—Ho1—O4	61.54 (11)	O1—C7—C6	124.6 (5)
O6—Ho1—O4	106.10 (14)	C2—C7—C6	119.1 (5)
O11—Ho1—O4	76.52 (13)	N1—C8—C6	126.2 (5)
O8—Ho1—O4	118.41 (12)	N1—C8—H8	116.9
O12—Ho1—O4	75.69 (14)	C6—C8—H8	116.9
O9—Ho1—O4	69.45 (12)	N2—C10—C9	109.0 (5)
O1—Ho1—O3	62.03 (12)	N2—C10—H10A	109.9
O2—Ho1—O3	127.20 (12)	C9—C10—H10A	109.9
O6—Ho1—O3	105.25 (14)	N2—C10—H10B	109.9
O11—Ho1—O3	75.75 (13)	C9—C10—H10B	109.9
O8—Ho1—O3	67.95 (12)	H10A—C10—H10B	108.3
O12—Ho1—O3	75.82 (14)	C7—C6—C5	118.5 (6)
O9—Ho1—O3	118.46 (12)	C7—C6—C8	123.4 (5)
O4—Ho1—O3	148.63 (12)	C5—C6—C8	117.8 (5)
O5—Zn1—O1	102.49 (16)	O4—C18—H18A	109.5
O5—Zn1—N2	110.09 (18)	O4—C18—H18B	109.5
O1—Zn1—N2	147.12 (18)	H18A—C18—H18B	109.5
O5—Zn1—O2	104.16 (16)	O4—C18—H18C	109.5
O1—Zn1—O2	78.64 (14)	H18A—C18—H18C	109.5
N2—Zn1—O2	89.09 (16)	H18B—C18—H18C	109.5
O5—Zn1—N1	112.60 (18)	C4—C5—C6	121.1 (6)
O1—Zn1—N1	89.23 (17)	C4—C5—H5	119.5
N2—Zn1—N1	82.44 (19)	C6—C5—H5	119.5
O2—Zn1—N1	143.00 (18)	C5—C4—C3	120.8 (6)
C7—O1—Zn1	126.1 (3)	C5—C4—H4	119.6
C7—O1—Ho1	130.6 (3)	C3—C4—H4	119.6
Zn1—O1—Ho1	101.65 (15)	C16—C15—C14	118.9 (6)
N5—O12—Ho1	94.7 (3)	C16—C15—H15	120.5
C17—O2—Zn1	127.8 (3)	C14—C15—H15	120.5
C17—O2—Ho1	131.3 (3)	N1—C9—C10	110.3 (5)
Zn1—O2—Ho1	100.93 (15)	N1—C9—H9A	109.6
C16—O4—C18	116.2 (4)	C10—C9—H9A	109.6
C16—O4—Ho1	118.3 (3)	N1—C9—H9B	109.6
C18—O4—Ho1	125.5 (3)	C10—C9—H9B	109.6
O2—C17—C12	125.0 (5)	H9A—C9—H9B	108.1
O2—C17—C16	115.3 (5)	C13—C14—C15	121.0 (6)
C12—C17—C16	119.7 (5)	C13—C14—H14	119.5
N4—O8—Ho1	96.9 (3)	C15—C14—H14	119.5
O10—N4—O9	122.4 (5)	C14—C13—C12	121.8 (6)
O10—N4—O8	122.1 (5)	C14—C13—H13	119.1
O9—N4—O8	115.4 (5)	C12—C13—H13	119.1
N3—O6—Ho1	144.0 (4)	C2—O3—C1	116.6 (4)
C2—C3—C4	118.8 (6)	C2—O3—Ho1	117.3 (3)
C2—C3—H3	120.6	C1—O3—Ho1	125.8 (3)
C4—C3—H3	120.6	O3—C1—H1A	109.5
O13—N5—O11	122.6 (5)	O3—C1—H1B	109.5
O13—N5—O12	120.9 (6)	H1A—C1—H1B	109.5
O11—N5—O12	116.5 (5)	O3—C1—H1C	109.5
N3—O5—Zn1	119.1 (3)	H1A—C1—H1C	109.5
O4—C16—C15	126.0 (5)	H1B—C1—H1C	109.5
O4—C16—C17	113.3 (5)		

### Hydrogen-bond geometry (Å, °)

**Table:**

*D*—H···*A*	*D*—H	H···*A*	*D*···*A*	*D*—H···*A*
C1—H1B···O11	0.96	2.54	3.167 (8)	123
C5—H5···O11^i^	0.93	2.45	3.377 (7)	174
C10—H10A···O13^ii^	0.97	2.54	3.483 (8)	165
C18—H18B···O9	0.96	2.58	3.100 (8)	114

Symmetry codes: (i) *x*−1/2, −*y*+1/2, *z*+1/2; (ii) −*x*+1, −*y*, −*z*+2.
